The article "circRNA_0001679/miR-338-3p/DUSP16 axis aggravates acute lung injury" was retracted in 2023. Reasons: duplicated images; concerns about the data; concerns about the images; concerns about a third party's involvement.

# circRNA_0001679/miR-338-3p/DUSP16 axis aggravates acute lung injury

**DOI:** 10.1515/med-2022-0417

**Published:** 2022-02-28

**Authors:** Jiang Zhu, Fukuan Zhong, Futao Chen, Yang Yang, Yingying Liao, Lifeng Cao, Yong Zhou, Qiaohong Bai

**Affiliations:** Department of Respiratory, The Second People’s Hospital of Lianyungang, Lianyungang 222023, Jiangsu, China; Department of Respiratory, The Second Hospital of Nanjing, Nanjing University of Chinese Medicine, Zhongfu Road 1, Gulou District, Nanjing 210003, Jiangsu, China

**Keywords:** circ_0001679, miR-338-3p, DUSP16, sepsis

## Abstract

Acute lung injury (ALI) is a respiratory disorder characterized by acute respiratory failure. circRNA mus musculus (mmu)-circ_0001679 was reported overexpressed in septic mouse models of ALI. Here the function of circ_0001679 in sepsis-induced ALI was investigated. *In vitro* models and animal models with ALI were, respectively, established in mouse lung epithelial (MLE)-12 cells and C57BL/6 mice. Pulmonary specimens were harvested for examination of the pathological changes. The pulmonary permeability was examined by wet-dry weight (W/D) ratio and lung permeability index. The levels of tumor necrosis factor (TNF)-α, interleukin (IL)-6, and IL-1β in the bronchoalveolar lavage fluid (BALF), the lung tissues, and the supernatant of MLE-12 cells were measured by enzyme linked immunosorbent assay . Apoptosis was determined by flow cytometry. Bioinformatics analysis and luciferase reporter assay were used to assess the interactions between genes. We found that circ_0001679 was overexpressed in lipopolysaccharide (LPS)-stimulated MLE-12 cells. circ_0001679 knockdown suppressed apoptosis and proinflammatory cytokine production induced by LPS. Moreover, circ_0001679 bound to mmu-miR-338-3p and miR-338-3p targeted dual-specificity phosphatases 16 (DUSP16). DUSP16 overexpression reversed the effect of circ_0001679 knockdown in LPS-stimulated MLE-12 cells. Furthermore, circ_0001679 knockdown attenuated lung pathological changes, reduced pulmonary microvascular permeability, and suppressed inflammation in ALI mice. Overall, circ_0001679 knockdown inhibits sepsis-induced ALI progression through the miR-338-3p/DUSP16 axis.

## 1 Introduction

Sepsis is a complex inflammatory disorder induced by bacterial infection, resulting in multi-organ dysfunction syndrome, including lung, kidney, liver, and cardiovascular system [1,2]. Acute lung injury (ALI) characterized by overwhelming hyperinflammation in lung is a severe complication of sepsis, with a high incidence and mortality [3]. Approximately 50% of patients with sepsis develop ALI [4,5]. Despite improved therapeutic strategies in clinical treatment for ALI, it is still a major challenge, with a mortality rate as high as 35–40% [6]. It is urgent to seek effective therapeutic biomarkers to improve the outcome of the disease. It has been reported that sepsis-induced ALI is related to alveolar epithelial cell apoptosis, abnormal inflammatory response in the lung, and excessive oxidative stress [7]. Inflammatory mediators and cytokines have been considered to play key roles in initiating, augmenting, and maintaining sepsis-induced ALI [8]. Studies show that the administration of lipopolysaccharide (LPS) has been widely used to establish sepsis-associated lung injury models [9].

The article "circRNA_0001679/miR-338-3p/DUSP16 axis aggravates acute lung injury" was retracted in 2023. Reasons: duplicated images; concerns about the data; concerns about the images; concerns about a third party's involvement.

Circular RNAs (circRNAs) are a group of noncoding RNAs that contribute to the pathophysiological process of diseases [10,11]. It has been reported that circRNAs exert vital functions on inflammatory response in ALI progression by regulating production of pro-inflammatory cytokines [12,13]. Furthermore, previous research showed the function of circRNAs in sepsis-related ALI. Li et al. showed significantly changed circRNA profiles in LPS‐induced mouse model and revealed a potential role of circRNAs in ALI [14]. Dysregulation of numerous circRNAs was found in the pulmonary macrophages of septic mice [15]. Interestingly, mus musculus (mmu)-circ_0001679 (gene symbol: klhl2) was significantly reported to be upregulated in septic mouse models with ALI [16]. However, the biological function of circ_0001679 in sepsis-induced ALI progression remains unclear. Moreover, circRNAs can act as microRNA (miRNA) “sponges” and upregulate the target gene by isolating and competitively inhibiting miRNA activity [17], thereby modulating progression of diseases [18,19,20]. We intended to explore whether circ_0001679 exerts its function in sepsis-induced ALI in such manner.

In this study, the function and molecular mechanisms of circ_0001679 in cell models of ALI by LPS stimulation were explored. Additionally, we examined the circ_0001679 expression and explored the effect of circ_0001679 on injury and inflammation in murine septic models with ALI. Our research may provide a potential insight for clinical treatment of sepsis-induced ALI.

## 2 Materials and methods

### 2.1 Animals and grouping

A total of 48 7-week-old C57BL/6 mice (male) were obtained from Vital River Co. Ltd (Beijing, China). Our experiments were approved by the Animal Ethics Committee of The Second Hospital of Nanjing, Nanjing University of Chinese Medicine. Animals were housed in groups of 5 per cage under 12 h light/12 h dark cycle at a temperature of 20 ± 2°C and 60–70% humidity. Food and water were available ad libitum. All delivered mice were kept for 1 week as an acclimatization period prior to performing any experiments. The mice were randomized into four groups: sham, ALI, ALI + adeno-associated virus (AAV)-sh-NC, and ALI + AAV-sh-circ_0001679 at random (*n* = 12 per group). To establish a mouse model with ALI, the mice were anesthetized and then intratracheally injected with 5 mg/kg LPS (Sigma-Aldrich, USA) in 50 µL of phosphate-buffered saline (PBS) [21]. The sham mice received the same dose of PBS. After 24 h, the mice were euthanized by 50 mg/kg pentobarbital (Sigma-Aldrich) through intraperitoneal injection. Seven days before LPS administration, the mice were intratracheally injected with 50 µL of PBS containing 5 × 10^10^ vector genomes of rAAV6-sh-circ_0001679 or rAAV6-sh-NC (all from Hanheng Company, Shanghai, China) under the effect of anesthesia.


The article "circRNA_0001679/miR-338-3p/DUSP16 axis aggravates acute lung injury" was retracted in 2023. Reasons: duplicated images; concerns about the data; concerns about the images; concerns about a third party's involvement.

**Ethical approval**: The experimental procedure was conducted in accordance with the Guidelines for the Care and Use of Laboratory Animals and approved by the Ethics Committee of The Second Hospital of Nanjing, Nanjing University of Chinese Medicine.

### 2.2 Cells

Mouse lung epithelial cells (MLE-12) were obtained from the American Type Culture Collection (ATCC; VA, USA), and cultured in Dulbecco’s Modified Eagle Medium (DMEM; Gibco, CA, USA) containing 10% FBS (Gibco), 100 mg/mL streptomycin, and 100 U/mL penicillin in a humidified environment at 37°C with 5% CO_2_. To induce inflammatory response, MLE-12 cells were treated with 10 ng/mL LPS for 48 h. The control cells were treated with the same dose of PBS.

### 2.3 Cell transfection

GenePharma Co., Ltd (Shanghai, China) designed and synthesized the plasmids used in this study. LPS-stimulated MLE-12 cells were seeded into 12-well plates at 2 × 10^5^ cells/well before the transfection. When cells reached approximately 80% confluence, they were transfected with miR-338-3p mimics (100 nM), NC mimics (100 nM), sh-NC (50 nM), and sh-circ_0001679 (50 nM). The sequence of dual-specificity phosphatase 16 (DUSP16) was constructed and inserted into the pcDNA3.1 (Invitrogen, USA) plasmids to generate pcDNA3.1/DUSP16. All transfections were performed using Lipofectamine 3000 (Invitrogen). Cells were incubated in serum-free medium for 6 h and then in DMEM containing serum for 48 h. Reverse transcription-quantitative polymerase chain reaction (RT-qPCR) was used to assess the transfection efficiency.

### 2.4 RT-qPCR

Total RNA was extracted from mouse lung tissues or MLE-12 cells using TRIzol (Invitrogen) following the manufacturer’s protocol and then reverse transcribed into cDNA by using the ReverTra Ace qPCR RT Kit (Toyobo, Japan) or the microRNA Reverse Transcription Synthesis Kit (Thermo Fisher Scientific, USA). Next PCR analysis was performed using the SYBR Premix Ex Taq II (Takara) on 7300 Real-time PCR System (Applied Biosystems, USA). The relative quantification was conducted using the 2^−ΔΔCt^ method. GAPDH or U6 served as internal references.

The article "circRNA_0001679/miR-338-3p/DUSP16 axis aggravates acute lung injury" was retracted in 2023. Reasons: duplicated images; concerns about the data; concerns about the images; concerns about a third party's involvement.

### 2.5 Western blot

Total proteins were separated with RIPA buffer (Roche, USA), sonicated, and centrifuged. Protein concentration was quantified using the Bicinchoninic Acid Assay Kit (Beyotime, Shanghai, China). Proteins were separated by 12% sodium dodecyl sulfate polyacrylamide gel and transferred to polyvinylidene fluoride membranes (Millipore, USA). Afterwards, the membranes were blocked with 5% skimmed milk for 1 h and were incubated with primary antibodies DUSP16 (ab181088, 1:1,000), Bcl-2 (ab182858, 1:2,000), Bax (ab182733, 1:2,000), and GAPDH (ab9485, 1:2,000) at 4°C overnight. Next day, second antibody horseradish peroxidase-labeled IgG was added and incubated for 2 h at 4°C. After washing, the Enhanced Chemiluminescent Kit (GE Healthcare Bio-Sciences, Pittsburgh, PA, USA) was utilized to visualize the proteins. Protein bands were detected using Image Lab Touch 3.0 Software (Bio-Rad, Hercules, USA).

### 2.6 Hematoxylin and eosin staining

The mouse lung samples of sham and model groups were removed and fixed with 4% paraformaldehyde for 48 h. The tissues were then dehydrated with graded concentrations of ethanol solution, permeabilized with xylene, embedded in paraffin, and then cut into 4 µm thick sections. Afterwards, the sections were dewaxed, hydrated, and stained with hematoxylin–eosin staining. The stained sections were then mounted in neutral balsam. The morphological changes were observed with a microscope (TE2000U; Nikon, Japan). The lung tissue damage was quantified using the lung tissue injury scoring (0: normal to 3: severe), including alveolar wall edema, hemorrhage, vascular congestion, and polymorphonuclear leukocyte infiltration. Lung injury was categorized according to the sum of the score (0–3: normal to minimal; 4–6: mild; 7–9: moderate; 10–12: severe inflammation), as previously reported [22].

### 2.7 Wet-to-dry weight (W/D) ratio

At the end of the experiment, the right lung was immediately removed. A portion of lung tissue from each animal was placed in a dry plastic boat and weighed (wet weight) with a precision scale. The tissue was then dried in an incubator at 60°C for 5 days and weighed again (dry weight). The W/D ratio was calculated as the ratio of the wet weight to the final dry weight as described elsewhere [23].

### 2.8 Lung permeability index

Plasma supernatants were obtained and stored at −70°C for determination of total plasma protein. After incision of the trachea, a plastic cannula was inserted, and airspaces were washed using 1 mL of saline (4 times with 0.25 mL). The BALF samples were then centrifuged (1,000 × *g* for 5 min) at room temperature, and supernatants were collected. BALF supernatant was then stored at −70°C for the detection of total BALF protein concentration using the Bradford protein concentration assay. Lung permeability index (LPI) was calculated by dividing BALF protein concentration by plasma protein concentration.

The article "circRNA_0001679/miR-338-3p/DUSP16 axis aggravates acute lung injury" was retracted in 2023. Reasons: duplicated images; concerns about the data; concerns about the images; concerns about a third party's involvement.

### 2.9 Enzyme linked immunosorbent assay (ELISA)

The levels of tumor necrosis factor (TNF)-α, interleukin (IL)-6, and IL-1β in the BALF, the lung tissues, and the supernatant of MLE-12 cells were detected by Mouse TNF-α ELISA Kit (cat. no. PT512; Beyotime), Mouse IL-6 ELISA Kit (cat. no. PI326; Beyotime), and Mouse IL-1β ELISA Kit (cat. no. PI301; Beyotime) according to the instructions, respectively. A Power Wave Microplate Reader (Bio-TEK, USA) was used to measure the absorbance at 450 nm.

### 2.10 Flow cytometry

An Annexin V-FITC/PI Apoptosis Detection Kit (Abcam, USA) was used. Briefly, after washing with cold PBS, the transfected MLE-12 cells in 6-well plates (1 × 10^5^ cells/well) were resuspended in annexin-binding buffer. Next 10 µL of PI and 5 µL of Annexin V-FITC were added and incubated with cells for 10 min at room temperature in the dark. Apoptotic cells were detected using a flow cytometer (BD Biosciences, USA), and the data were analyzed using FlowJo software (TreeStar, CA, USA).

### 2.11 Luciferase reporter assay

The wild-type (WT) binding sequence of circ_0001679 or DUSP16 3′-UTR on miR-338-3p was inserted into the pmirGLO luciferase vector to construct pmirGLO-circ_0001679-WT or pmirGLO-DUSP16-WT plasmids. The mutant (Mut) sequence of circ_0001679 or DUSP16 in miR-338-3p was inserted in the same way. These plasmids were co-transfected into MLE-12 cells with miR-338-3p mimics or NC mimics using Lipofectamine 3000. After 48 h, the luciferase activity of each group was assessed using the Dual Luciferase Kit (Promega, USA)

### 2.12 Statistical analysis

All data from three independent experiments are shown as the mean value ± standard deviation (SD). Student’s *t* test was applied for statistical analysis of two groups and one-way analysis of variance was applied for statistical analysis of multiple groups (not less than three groups). All data were processed with SPSS 20.0 Software (SPSS Inc., USA). The correlation between gene expressions in mouse lung tissues was analyzed by Pearson correlation analysis. The value of *p* < 0.05 was statistically significant.

## 3 Results

### 3.1 Circ_0001679 knockdown inhibits MLE-12 cell apoptosis and inflammation

First, circ_0001679 expressions in MLE-12 cells upon LPS stimulation were determined. The RT-qPCR results showed that circ_0001679 expression in LPS-stimulated MLE-12 cells was higher than that in the control cells (Figure 1a). Subsequently, circ_0001679 was knocked down by transfection with sh-circ_0001679 into MLE-12 cells (Figure 1b). The concentrations of proinflammatory cytokines were assessed using ELISA. It was shown that LPS stimulated the production of IL-1β, IL-6, and TNF-α, and circ_0001679 knockdown attenuated this effect (Figure 1c–e). In addition, flow cytometry analysis showed that the apoptosis of MLE-12 cells was promoted after LPS treatment and was further inhibited by circ_0001679 knockdown (Figure 1f). Furthermore, western blot analysis showed that an increase in Bax protein level and a decrease in Bcl-2 protein level were caused by LPS and then reversed by circ_0001679 downregulation (Figure 1g).

The article "circRNA_0001679/miR-338-3p/DUSP16 axis aggravates acute lung injury" was retracted in 2023. Reasons: duplicated images; concerns about the data; concerns about the images; concerns about a third party's involvement.

**Figure 1:** Circ_0001679 knockdown inhibits cell apoptosis and inflammation. (a and b) RT-qPCR analysis of circ_0001679 expression in MLE-12 cells under the indicated treatment. (c–e) ELISA of the concentrations of IL-1β, IL-6, and TNF-α in MLE-12 cells under the indicated treatment. (f) Flow cytometry analysis of the apoptosis of MLE-12 cells under the indicated treatment. (g) Western blot analysis of the Bax and Bcl-2 protein levels in MLE-12 cells under the indicated treatment. Data are shown as the mean value ± SD. The experiments were repeated three times. *p < 0.05, **p < 0.01, and ***p < 0.001.

### 3.2 Circ_0001679 binds to miR-338-3p

We then aimed to investigate the circ_0001679-mediated molecular mechanisms in MLE-12 cells. circRNAs can competitively bind to microRNAs (miRNAs) to release the activity of messenger RNAs (mRNAs) [24,25,26]. By examining starBase database (http://starbase.sysu.edu.cn/), we found ten miRNAs that have binding sites for circ_0001679. RT-qPCR indicated that mmu-miR-338-3p was significantly downregulated in LPS-treated MLE-12 cells compared to the other miRNAs (Figure 2a). RT-qPCR indicated that the miR-338-3p level was elevated by transfection with miR-338-3p mimics (Figure 2b). The binding site between circ_0001679 (chr8:64811729-64811750[-]) and miR-338-3p was predicted in starBase (Figure 2c). We mutated the WT binding sequence of miR-338-3p in circ_0001679 and then performed luciferase reporter assay. Overexpression of miR-338-3p eliminated the luciferase activity of circ_0001679-WT reporters and did not affect that of circ_0001679-Mut reporters (Figure 2d), demonstrating the binding affinity of circ_0001679 to miR-338-3p.

**Figure 2:** Circ_0001679 binds to miR-338-3p. (a) RT-qPCR analysis of the expression of candidate miRNAs in LPS-treated MLE-12 cells. (b) RT-qPCR analysis of the transfection efficiency of miR-338-3p mimics in MLE-12 cells. (c) The binding site of miR-338-3p in circ_0001679 (chr8:64811729-64811750[−]) predicted in starBase. (d) Luciferase reporter assay of the binding ability of miR-338-3p to circ_0001679. Data are shown as the mean value ± SD. The experiments were repeated three times. *p < 0.05, **p < 0.01, and ***p < 0.001.

The article "circRNA_0001679/miR-338-3p/DUSP16 axis aggravates acute lung injury" was retracted in 2023. Reasons: duplicated images; concerns about the data; concerns about the images; concerns about a third party's involvement.

### 3.3 DUSP16 is targeted by miR-338-3p

From the miRDB database (http://mirdb.org/), we found 5 potential targets of miR-338-3p (predicted binding scores over 96). The RT-qPCR results suggested that DUSP16 was significantly upregulated in LPS-stimulated MLE-12 cells, and the expression levels of other candidates showed no significant change (Figure 3a). Therefore, DUSP16 was chosen for further research. In Figure 3b, the putative binding sequence of miR-338-3p in DUSP16 was found in TargetScan (http://www.targetscan.org/vert_70/), which is highly conserved in multiple species. The WT binding sequence of miR-338-3p in DUSP16 3′-UTR was mutated. The luciferase activity of DUSP16 3′-UTR-WT reporters was notably decreased in response to miR-338-3p overexpression, and that of DUSP16 3′-UTR-Mut reporter showed no significant change in MLE-12 cells (Figure 3c). It suggested that miR-338-3p directly targets DUSP16. Furthermore, the DUSP16 protein level was reduced after circ_0001679 knockdown or miR-338-3p overexpression (Figure 3d).

**Figure 3:** DUSP16 is targeted by miR-338-3p. (a) RT-qPCR analysis of the expression of candidate targets in LPS-treated MLE-12 cells. (b) The binding site of miR-338-3p in DUSP16 3'-UTR predicted in TargetScan. (c) Luciferase reporter assay of the binding ability of miR-338-3p to DUSP16. (d) Western blot analysis of the DUSP16 protein level in MLE-12 cells under the indicated transfection. Data are shown as the mean value ± SD. The experiments were repeated three times. **p < 0.01 and ***p < 0.001.

### 3.4 Circ_0001679 promotes cell apoptosis and inflammation by upregulating DUSP16

We intended to explore whether DUSP16 participates in the circ_0001679-mediated regulation of LPS-stimulated MLE-12 cells. Western blot demonstrated the upregulation of DUSP16 expression in MLE-12 cells after transfection with pcDNA3.1/DUSP16 (Figure 4a). Moreover, DUSP16 overexpression reversed the decreased concentrations of cytokines under circ_0001679 knockdown in LPS-stimulated MLE-12 cells (Figure 4b–d). Additionally, DUSP16 overexpression prevented the suppressive effect of circ_0001679 knockdown on the apoptosis of LPS-stimulated MLE-12 cells (Figure 4e). Furthermore, the change in Bax and Bcl-2 protein levels induced by circ_0001679 knockdown was reversed by DUSP16 overexpression (Figure 4f).

The article "circRNA_0001679/miR-338-3p/DUSP16 axis aggravates acute lung injury" was retracted in 2023. Reasons: duplicated images; concerns about the data; concerns about the images; concerns about a third party's involvement.

**Figure 4:** Circ_0001679 promotes cell apoptosis and inflammatory response by upregulating DUSP16. (a) Western blot analysis of DUSP16 expression in MLE-12 cells after transfection with pcDNA3.1/DUSP16. (b–d) ELISA of the concentrations of IL-1β, IL-6, and TNF-α in MLE-12 cells under the indicated treatment. (e) Flow cytometry analysis of the apoptosis of MLE-12 cells under the indicated treatment. (f) Western blot analysis of the Bax and Bcl-2 protein levels in MLE-12 cells under the indicated treatment. Data are shown as the mean value ± SD. The experiments were repeated three times. *p < 0.05, **p < 0.01, and ***p < 0.001.

### 3.5 Circ_0001679 knockdown alleviates lung injury in ALI mice

To further investigate the function of circ_0001679 *in vivo*, murine septic models with ALI induced by LPS administration were established. Hematoxylin and eosin staining showed that LPS resulted in significant inflammatory infiltration, alveolar structure destruction, and pulmonary edema in the lung tissues, which could be obviously ameliorated after AAV-sh-circ_0001679 injection (Figure 5a). Similarly, AAV-sh-circ_0001679 significantly reduced the increased lung injury score in the ALI group (Figure 5b). Increased pulmonary permeability led to pulmonary edema. In the present study, we assessed the extent of pulmonary edema by W/D ratio and lung permeability index. Compared with the sham group, W/D ratio and lung permeability index were increased in the ALI group. AAV-sh-circ_0001679 significantly decreased W/D ratio and lung permeability index (Figure 5c and d). These findings indicated that silencing circ_0001679 decreases epithelial barrier permeability and alleviates pulmonary edema. Moreover, obvious increase in concentrations of IL-1β, IL-6, and TNF-α in the BALF and the lung tissues of ALI mice was observed. However, AAV-sh-circ_0001679 injection effectively restrained the above changes (Figure 5e–g). Furthermore, the change in the protein levels, Bax and Bcl-2, in the lung tissues of ALI mice was reversed by AAV-sh-circ_0001679 (Figure 5h). RT-qPCR analysis showed that circ_0001679 and DUSP16 were upregulated and miR-338-3p was downregulated in ALI mouse lung tissues. After injection with AAV-sh-circ_0001679, the circ_0001679 and DUSP16 expression levels were reduced (Figure 5i–k). Meanwhile, DUSP16 expression was positively correlated with circ_0001679 expression in ALI mouse lung tissues (Figure 5l), and, in parallel, DUSP16 expression or circ_0001679 expression was negatively associated with miR-338-3p expression (Figure 5m and n).

The article "circRNA_0001679/miR-338-3p/DUSP16 axis aggravates acute lung injury" was retracted in 2023. Reasons: duplicated images; concerns about the data; concerns about the images; concerns about a third party's involvement.

**Figure 5:** Circ_0001679 knockdown alleviates lung injury and reduces inflammation in ALI mice. (a) The histological changes in lungs of ALI mice and sham mice were analyzed by hematoxylin and eosin staining. (b) Lung injury scores were analyzed and recorded. (c) Lung W/D ratio of mice and (d) lung permeability index in the lung tissues. (e–g) ELISA of the concentrations of IL-1β, IL-6, and TNF-α in the BALF and the lung tissues in each group. (h) Western blot analysis of the Bax and Bcl-2 protein levels in the lung tissues in each group. RT-qPCR analysis of (i) circ_0001679 expressions, (j) DUSP16 expression, and (k) miR-338-3p expression in the lung tissues in each group. (l–n) Pearson correlation analysis of the expression relationship between circ_0001679, DUSP16, and miR-338-3p in ALI mouse lung tissues. *N* = 12 per group. Data are shown as the mean value ± SD. The experiments were repeated three times. *p < 0.05, **p < 0.01, and ***p < 0.001.

## 4 Discussion

Accumulating research has revealed that abnormal production of inflammation cytokines is a key event in sepsis-induced ALI [27,28]. In our study, we used LPS to establish MLE-12 cell models to mimic the characteristics of sepsis-induced ALI. LPS significantly promoted proinflammatory cytokine production and apoptosis in MLE-12 cells. It has been revealed that mmu-circ_0001679 expression is upregulated in septic mouse models with ALI [16]. Here circ_0001679 was upregulated in LPS-treated MLE-12 cells and lung tissues of ALI mice. Functionally, circ_0001679 knockdown reversed the increased proinflammatory cytokine production and apoptosis. More importantly, circ_0001679 knockdown attenuated lung pathological changes, reduced pulmonary microvascular permeability, and suppressed inflammation in ALI mice. Therefore, we concluded that circ_0001679 may contribute to sepsis-induced ALI progression.

circRNAs can suppress mRNA degradation by sponging miRNAs through forming a ceRNA network [17]. For example, circTLK1 aggravates sepsis-induced ALI by augmenting oxidative stress and inflammation by the miR-106a-5p/HMGB1 axis [29]. circ_0091702 sponges miR-545-3p and upregulates THBS2 to mitigate sepsis-related ALI [30]. Additionally, numerous miRNAs were revealed to be involved in regulation of the inflammatory response in sepsis-induced ALI progression [31,32]. In our report, mmu-miR-338-3p was predicted to have a binding site for mmu-circ_0001679. MiRNA-338-3p was reported to prevent acute liver inflammation induced by acetaminophen in mice [33]. Additionally, miR-338-3p is downregulated in LPS-stimulated human bronchial epithelial cells and attenuates LPS-induced inflammation [34]. Here we found that the miR-338-3p level was reduced in LPS-stimulated MLE-12 cells and mouse models of sepsis-induced ALI. In addition, mechanical experiments confirmed that circ_0001679 bound to miR-338-3p, suggesting that circ_0001679 may regulate sepsis-induced ALI progression by interacting with miR-338-3p.

The article "circRNA_0001679/miR-338-3p/DUSP16 axis aggravates acute lung injury" was retracted in 2023. Reasons: duplicated images; concerns about the data; concerns about the images; concerns about a third party's involvement.

DUSP16, as a member of DUSPs family, could be inducible in macrophages [35]. It has been previously revealed that DUSP16 negatively regulates JNK pathway to attenuate metabolic stress-triggered hepatic steatosis [36]. Here bioinformatics analysis predicted that DUSP16 was a downstream gene of miR-338-3p. DUSP16 was upregulated in cell models of sepsis-induced ALI. Mechanistically, miR-338-3p targeted DUSP16 3′-UTR to reduce DUSP16 expression. Moreover, DUSP16 expression was negatively modulated by miR-338-3p and positively regulated by circ_0001679. Rescue assays validated that DUSP16 overexpression reversed the decreased proinflammatory cytokine production and apoptosis under circ_0001679 knockdown in LPS-treated MLE-12 cells.

In conclusion, we confirmed the upregulation of circ_0001679 and DUSP16 as well as downregulation of miR-338-3p in LPS-treated MLE-12 cells and ALI mouse lung tissues. We innovatively put forward and confirmed that circ_0001679 knockdown inhibits sepsis-induced ALI progression through reducing release of inflammation cytokines and inhibiting cell apoptosis *in vitro* and *in vivo* through the miR-338-3p/DUSP16 axis. Our research may provide a theoretical direction for treatment of sepsis-induced ALI.
